# The Regulatory Effect of Firm Size on Digital Transformation: An Empirical Study of Pharmaceutical Companies in China

**DOI:** 10.1155/2022/7731174

**Published:** 2022-10-03

**Authors:** Xiaowen Luo, Shun-Chi Yu

**Affiliations:** ^1^International College, National Institute of Development Administration, Bangkok 10240, Thailand; ^2^College of Applied Technology, Yunnan Minzu University, Kunming 650504, China

## Abstract

Digital transformation (DT) has been a key way for pharmaceutical companies to enhance innovation and R&D capabilities, improve product quality, reduce costs, and create competitive advantages. The external environment factors and the internal conditions' factors are the main factors affecting the DT of pharmaceutical companies. This research aimed to probe the effects of the external environment factors, the internal conditions' factors, firm size, and control variables on the DT of pharmaceutical companies based on synergetics. Purposive sampling and snowball sampling were used in this research. In addition, this research collected 395 valid data from Chinese pharmaceutical companies through online questionnaires. This research used quantitative analysis, and SPSS and Amos software were applied to data processing analysis. The results of structural equation modelling (SEM) and regression analysis showed that the external environment factors and the internal conditions' factors had a significantly positive correlation with the DT of pharmaceutical companies, and the effects of the internal conditions on the DT of pharmaceutical companies were greater than that of the external environment. In addition, firm size positively moderated the relationship between the external environment, internal conditions, and the DT of pharmaceutical companies. The results of this research not only can provide theoretical reference for scholars but also put forward implementation suggestions of DT for Chinese pharmaceutical company managers.

## 1. Introduction

China's pharmaceutical industry has developed rapidly, and the scale of China's pharmaceutical market has grown from RMB 955.5 billion in 2012 to RMB 2.15 trillion in 2020 [1]. However, problems such as weak innovation ability and weak competitiveness of China's pharmaceutical industry are prominent. In addition, the intensification of market competition has put forward higher requirements and challenges for operation management and cost control of pharmaceutical companies. Therefore, promoting the DT of pharmaceutical companies is an effective means to promote the transformation and upgrading of pharmaceutical companies to innovative technology and enhance their competitiveness. Macroeconomic factors leading to the DT of the pharmaceutical industry include technological innovation, new regulations, increased drug production costs, and new demands from users [2]. There are many factors that affect the DT of enterprises, which come from the external environment of the companies, including political, economic, technological, customer needs, and other factors [3]. There are factors from within the company's organization, including strategy, corporate culture, leadership, dynamic capabilities, organizational characteristics, innovation, and other factors [4]. If the main influencing factors of DT can be found and effective measures can be adopted to promote the DT of pharmaceutical companies, it is necessary to study the influencing factors of DT. Haken et al. [5] thought that greater effects can be generated through interaction between systems, often from external and internal collaboration. The application of digital technology can help companies to improve their internal cooperation ability [6]. However, DT is systematic and very complex, which requires multiparty cooperation, such as cooperation between government and companies, companies and companies, and companies and universities [7].

The aim of this research is to discover the main factors affecting the DT of pharmaceutical companies by reviewing the literature on the external environment, the internal conditions, firm size, control variables, and DT of pharmaceutical companies and to build the model of the factors affecting DT. Quantitative analysis was utilized to test the relationship between variables and DT through SEM and regression analysis. Finally, this research can integrate the factors that affect the DT of pharmaceutical companies and put forward the implementation suggestions of DT for pharmaceutical companies.

## 2. Literature Review and Research Hypotheses

### 2.1. The Factors of External Environment

Zhu et al. [8] considered that technological capabilities and competitive pressures can influence digital transformation. Tarutė et al. [3] thought that the digital transformation of small and medium-sized enterprises can be affected by external factors. Wilaisakoolyong [9] considered that digital technologies, costs reduction, productivity improvement, government policies, the upgrading of consumer behaviour, and pressure of market competition are the main factors affecting the digital transformation of companies. Hadia and Hmoodb [10] thought that the requirements of organization expansion, the pursuit of market share growth, and market competition are major reasons for the company to implement digital transformation. Tsenzharik et al. [11] thought that government policies can promote the digital transformation of companies. The relevant government departments should lay down financial support policies and special plans to support companies in implementing digital transformation projects, provide subsidies for those companies that apply digital technologies, and then promote the digitalization of companies [12]. It is necessary for the government to formulate relevant policies to regulate the digital transformation of enterprises, and the ICT infrastructures are the foundation of the digital transformation of enterprises [13]. Digital technology plays a role in ensuring digital transformation of enterprises [14]. Therefore, the above findings lead to the following assumptions.

  H1: The external environment can have a significant influence on the DT of pharmaceutical companies
  H1a: Customer needs can have a significant influence on the DT of pharmaceutical companies
  H1b: Market competition can have a significant influence on the DT of pharmaceutical companies
  H1c: Government policy can have a significant influence on the DT of pharmaceutical companies
  H1d: Digital technology can have a significant influence on the DT of pharmaceutical companies

### 2.2. The Factors of Internal Conditions

Factors within the organization's internal conditions can facilitate the digital transformation of companies [15, 16]. Kane et al. [17] considered that a digital strategy is the key to the success of business transformation. Agile and learning organizations support the digital transformation of companies [18]. Leadership's digital awareness can affect an organization's digital transformation [19]. Senior leadership's support for digital transformation can determine the success or failure of a company's digital transformation [20]. Therefore, the above findings lead to the following assumptions.

  H2: The internal conditions can have a significant influence on the DT of pharmaceutical companies
  H2a: Digital strategy can have a significant influence on the DT of pharmaceutical companies
  H2b: Organization capability can have a significant influence on the DT of pharmaceutical companies
  H2c: Leadership can have a significant influence on the DT of pharmaceutical companies

### 2.3. Firm Size

The firms can be divided into different scales according to the number of employees, income, and total assets. The division standard of firm size in different industries is different. The number of employees of the company can affect whether the company carries out the DT projects. Firm size and its capabilities can affect the success of digital transformation [21, 22]. Firm size can influence the urgency of digital transformation [23]. Firm size has a regulatory effect in artificial intelligence applications on the performance of manufacturing firms [24]. Larger companies are more experienced in management and have more capital, human resources, digital skills, and relatively strong capabilities to advance digitalization. Firm size plays a role in the DT of companies. This study mainly divides firm size based on the number of employees. Therefore, the above findings lead to the following assumptions.

  H3: Firm size can have a significantly regulatory influence on the relationship between the external environment and the DT of pharmaceutical companies
  H4: Firm size can have a significantly regulatory influence on the relationship between the internal conditions and the DT of pharmaceutical companies

### 2.4. The Control Variables

The ownership types of Chinese enterprises include state-owned enterprises and private enterprises [25]. Eller et al. [26] considered that the type of ownership and the age of the company have positive effects on the DT of SMEs. The region, industry, and the age and business volume growth of the company can affect the transformation and upgrading of manufacturing companies [27, 28]. Senior leaders play a decisive role in the digital transformation of companies [29]. The current DT situation of companies can affect the implementation of DT in the next step [30]. Therefore, this research selected five control variables, including staff position, the region which the company belongs to, the age of the company, the type of company ownership, and the DT situation of the company.

### 2.5. Research Framework

From the research results of previous scholars, it was concluded that the external environmental factors and the internal conditions' factors were the main factors affecting the DT of pharmaceutical companies [31], and firm size played a regulatory role in the DT of pharmaceutical companies. According to literature, this research formed the related theoretical framework, as shown in Figure 1.

## 3. Methods

### 3.1. Sample and Data Collection

Since the implementation of pharmaceutical companies' DT required a high degree of professionalism, the sample objects of this research were mainly general staff, the first-line managers, and middle managers and senior managers of pharmaceutical companies.

Purposive sampling focused on candidates with similar characteristics or specific characteristics related to the subject being studied [32]. Snowball sampling pointed at the selection and investigation of several people with the characteristics required for research purposes, relying on them to select people who met the needs of the research [33]. In order to ensure the representativeness of the sample, purposive sampling and snowball sampling were applied to collect data through online questionnaires. From April 10 to May 15, 2022, a number of pharmaceutical companies in various provinces in China sent out questionnaires, and a total of 443 questionnaires were recovered, and 395 questionnaires were valid, and the validity rate reached 89.16%.

The descriptive statistics for the questionnaire were shown in Table 1. The distribution of the region which the sample belongs to was discrete, and the distribution of the sample objects was a normal distribution, which had good external validity. According to the type of company ownership, a number of state-owned enterprises were 149, accounting for 37.72%. A number of private enterprises were 246, accounting for 62.28%. According to the situation of pharmaceutical companies' DT, pharmaceutical companies that have not undergone DT and have no willingness and plan for DT accounted for 6.33%; pharmaceutical companies that have not undergone DT and have DT willingness and plans accounted for 16.71%; pharmaceutical companies that have undergone DT and whose DT projects are in the early stages of construction accounted for 30.63%; and pharmaceutical companies that have undergone DT and have achieved certain results in DT projects accounted for 46.33%. It can be seen that DT is the general development trend for pharmaceutical companies of China.

### 3.2. Measures

This questionnaire was compiled on the basis of the measurement scale used in previous studies, and the scale had been validated by other scholars. The Likert scale and five subjective measures were applied in this research [34]. The external environment scale was mainly composed of customer needs, market competition, government policy, and digital technology [31]. The scale of the customer needs consisted of five measurement items, such as “Do you think the improvement of customer spending power has an important influence on DT?” The scale of market competition was composed of five measurement items, such as “Do you think market competition pressure in the same industry has an important influence on DT?” The scale of government policy was composed of four measurement items, such as “Do you think government financial support and incentives have an important influence on DT?” The scale of digital technology was composed of four measurement items, such as “Do you think the support of information infrastructure has an important influence on DT?” The internal condition scale mainly consisted of digital strategy, organization capability, and leadership [31]. The scale of digital strategy was composed of four measurement items, such as “Do you think developing a digital strategy has an important influence on DT?” The scale of organization capability was composed of six measurement items, such as “Do you think organization agility has an important influence on DT?” The leadership scale was composed of four measurement items, such as “Do you think leadership awareness has an important influence on DT?” The scale of company DT was composed of four measurement items, such as “Do you think company DT will drive organization transformation?”

## 4. Results Analysis

### 4.1. Reliability Analysis

SPSS 25.0 was used for reliability analysis in this research. Tavakol and Dennick [35] considered that the corrected-item total correlation (CITC) value of each dimension exceeds 0.5, and the Cronbach's alpha value exceeds 0.7, indicating that the scale has high reliability. Cronbach [36] deemed that when the CITC value of a scale item is less than 0.5, and the item should be deleted. According to the reliability analysis results, it can be seen that the external environmental variables were measured through customer needs, market competition, government policy, and digital technology [31]. The CITC value of CN1 in the customer needs dimension was less than 0.5, and the overall reliability of customer needs after CN1 was deleted had increased from 0.695 to 0.822; the CITC value of MC4 in the market competition dimension was less than 0.5, and the overall reliability of market competition after when MC4 was deleted had increased from 0.887 to 0.916; the CITC value of GP3 in the government policy dimension was less than 0.5, and the overall reliability of government policies after GP3 was deleted had increased from 0.731 to 0.913; and the CITC value of TT2 in the digital technology dimension was less than 0.5, and the overall reliability of digital technology after TT2 was deleted had increased from 0.674 to 0.873. Therefore, after removing CN1, MC4, GP3, and TT2, the overall reliability of the external environment had increased from 0.880 to 0.916.

The internal condition variables were measured through digital strategy, organization capability, and leadership. The CITC values of OC2 and OC3 in the organization capability dimension were less than 0.5, and the overall reliability of organization capability after OC2 and OC3 which was deleted had increased from 0.723 to 0.881; the CITC value of LS2 in the leadership dimension was less than 0.5, and the overall reliability of leadership after LS2 was deleted had increased from 0.733 to 0.883. Therefore, after removing OC2, OC3, and LS2, the overall reliability of the internal condition had increased from 0.837 to 0.889. Therefore, after removing unreasonable items, the Cronbach's alpha of each dimension exceeded 0.7. It followed that the questionnaire scale used in this research had good reliability.

### 4.2. Validity Analysis

Confirmatory factor analysis is utilized to verify the validity of scales from three aspects: convergent validity, model fit, and discriminant validity. Factors such as factor loading, composite reliability (CR), and average variance extracted (AVE) are used to measure convergent validity. Factor loading reflects the degree to which measurement items can be applied to reflect latent variables, generally exceeding 0.5 [37]. CR exceeds 0.6, indicating that the internal quality of the model is ideal [38]. AVE reflects the convergence degree of a potential variable, which is required to exceed 0.5 [39]. The standardized factor loadings of each measurement item exceeded 0.5. As shown in Table 2, the CR of each variable exceeded 0.6, indicating that the intrinsic quality of each measurement scale was good. The AVE of each variable all exceeded 0.5. It can be concluded that the scale had good convergent validity.

Fornell and Larcker [40] deemed that the square root of each variable's AVE exceeds the correlation coefficient value of its column and row, indicating that the discriminant validity satisfies the analysis requirements. According to the results of Table 2, the measurement scale had good discriminant validity.

The operation of AMOS 23.0 had achieved the confirmatory factor model of the overall variables, the second-order factor model of the external environment factors, the second-order factor model of the internal conditions' factors, and the SEM model of DT. According to the results of Table 3, the fitting indices of each model met the general standard, indicating that the four measurement models had good fitting effects.

### 4.3. Correlation Analysis

Ong and Puteh [39] considered that the correlation test is applied to probe whether there is a certain correlation between variables. This research made use of Pearson's correlation to analyse the relationship between variables. The correlation analysis results are shown in Table 4.

On account of control variables, there was a positive correlation between staff position and DT (correlation coefficient (CC) = 0.169, *P* < 0.01); there was a negative correlation between the region of the company and DT (CC = −0.157, *P* < 0.05); the age of the company was positively related to DT (CC = 0.199, *P* < 0.01); the ownership type of the company was negatively related to DT (CC = −0.132, *P* < 0.01); and there was a positive correlation between the DT situation of the company and DT (CC = 0.138, *P* < 0.01). On account of moderating variables, there was a positive correlation between firm size and DT (CC = 0.216, *P* < 0.01). The expansion of firm size had a positive effect on DT. On account of independent variables, the external environment was positively related to DT (CC = 0.535, *P* < 0.01), and customer needs, market competition, government policy, and digital technology variables in the external environment were also positively related to DT. There was a positive correlation between the internal conditions and DT (CC = 0.573, *P* < 0.01), and digital strategy, organization capability, and leadership variables in the internal conditions were also positively related to DT.

In this research, AMOS 23.0 was used to verify the SEM model of the influencing factors of pharmaceutical companies' DT, and this model was used for parameter estimation and path analysis. The results are shown in Table 5 and Figure 2. The standardized path coefficient of the external environment on DT was 0.43 (*t* = 7.094, *P* < 0.001), indicating that the external environment had a significant influence on DT, so H1 is valid. The standardized path coefficient of the internal conditions on DT was 0.59 (*t* = 8.081, *P* < 0.001), indicating that the internal conditions have a significant influence on DT, so H2 is valid. In addition, since the standardized path coefficient of [IC-DT] was larger than that of [EE-DT], it showed that the influence of the internal conditions on the DT of pharmaceutical companies exceeded that of the external environment.

### 4.4. The Common Method Biases Test

The Harman single factor method was used in this research. As shown in Table 6, the nonrotating factor analysis showed that there were eight factors with characteristic roots exceeding 1, of which the factor with the largest characteristic root can explain 35.753% of the overall variation. There were no serious common method biases in the data of research [41].

### 4.5. Multicollinearity Test

When the tolerance exceeds 0.1 and the variance inflation factor (VIF) is less than 10, it indicates that there is no multicollinearity between variables [42]. The test of collinearity in this research found that the tolerance of each variable exceeded 0.1, and the VIF was less than 10, indicating that there was basically no multicollinearity between variables.

### 4.6. Regression Analysis

According to the results of Table 7, Model 1 used the control variables (position, region, age, type, and action) to perform regression analysis on the DT of the company. P3 (*β* = 0.303, *P* < 0.05) and P4 (*β* = 0.383, *P* < 0.001) indicated that the influence level of senior managers on the DT of the company was higher than that of general staff and middle managers; R2 (*β* = 0.251, *P* < 0.05) and R4 (*β* = −0.463, *P* < 0.001) indicated that regions with a high degree of economic development had a greater impact on the DT of the company; A3 (*β* = 0.503, *P* < 0.01) and A4 (*β* = 0.46, *P* < 0.05) indicated that the longer the company was established, the greater the impact on the DT of the company was; Action 2 (*β* = −0.628, *P* < 0.01), Action 3 (*β* = −0.449, *P* < 0.05), and Action 4 (*β* = −0.532, *P* < 0.05) indicated that the situation of “the company has not carried out DT, and has no willingness and plan for DT” had a significantly negative impact on the DT of the company. Therefore, the staff position, the region which the company belongs to, the age of the company, and the DT situation of the company had varying degrees of impact on the DT of the company. Model 2 reported the results of H1a, which supported a significantly positive relationship between customer needs and DT (*β* = 0.389, *P* < 0.001). Model 3 reported the results of H1b, which supported a significantly positive relationship between market competition and DT (*β* = 0.352, *P* < 0.001). Model 4 reported the results of H1c, which supported a significantly positive relationship between government policy and DT (*β* = 0.348, *P* < 0.001). Model 5 reported the results of H1d, which supported a significantly positive relationship between digital technology and DT (*β* = 0.331, *P* < 0.001). Model 7 reported the results of H3 (the *β* value of Zscore(Size) ∗ Zscore(EE) was 0.104, *P* < 0.01), and *R*^2^ had increased from 0.364 of Model 6 to 0.378, which confirmed that firm size positively moderated the relationship between the external environment and DT.

According to the results of Table 8, Model 9 reported the results of H2a, which supported a significantly positive relationship between digital strategy and DT (*β* = 0.297, *P* < 0.001). Model 10 reported the results of H2b, which supported a significantly positive relationship between organization capability and DT (*β* = 0.461, *P* < 0.001). Model 11 reported the results of H2c, which supported a significantly positive relationship between leadership and DT (*β* = 0.337, *P* < 0.001). Model 13 reported the results of H4 (the *β* value of Zscore(Size) ∗ Zscore(IC) was 0.092, *P* < 0.01), and *R*^2^ had increased from 0.369 of Model 12 to 0.38, which confirmed that firm size can positively moderate the relationship between the internal conditions and DT.

In conclusion, the hypotheses of this research were verified to be true according to the previous empirical evidence, as shown in Table 9.

## 5. Discussion

This research explored the relationship and effects of the external environment factors, the internal conditions' factors, firm size, and other control variables with the DT of pharmaceutical companies. The results of SEM and regression analysis can support all the proposed hypotheses. Firstly, the analysis of the results of the SEM model showed that the external environment factors can significantly affect the DT of pharmaceutical companies, which was in accordance with the previous research results [3, 8]. The internal conditions' factors can significantly affect the DT of pharmaceutical companies, which was in accordance with the previous research results [11, 15]. Particularly, this research found that the internal conditions' factors had a greater influence on pharmaceutical companies' DT than the external environment factors and provided additional support to previous research. Secondly, according to the regression analysis results, it was shown that firm size can positively moderate the relationship between the external environment factors, the internal conditions' factors, and the DT of pharmaceutical companies, which was in accordance with the previous research results [21]. In addition, senior managers can play a decisive role in the formulation and implementation of DT strategies, which was consistent with the previous research results [29].

## 6. Conclusion

In conclusion, the research provided empirical evidence for the influence of the external environment factors, the internal conditions' factors, and firm size on the DT of Chinese pharmaceutical companies. The external environment factors and the internal conditions' factors were significant factors affecting the DT of pharmaceutical companies, but the internal conditions' factors had a greater influence on DT. In addition, this research found that firm size can positively moderate the relationship between the external environment, the internal conditions, and pharmaceutical companies' DT. The larger the firm size was, the more urgent and influential the need for DT had. Therefore, pharmaceutical companies implemented DT projects according to their firm size and internal conditions. This research can fill the research gaps of pharmaceutical companies' DT by exploring the relationship and effects between the external environment, internal conditions, and firm size on pharmaceutical companies' DT and also put forward suggestions for promoting the DT implementation of pharmaceutical companies. Finally, pharmaceutical companies increasingly have realized that DT is a fast solution for companies to develop, and it is essential to explore the implementation paths of DT according to their own characteristics.

### 6.1. Theoretical and Practical Implications

The theoretical significance of this research is to build the model of the influencing factors of pharmaceutical companies' DT and confirm the influence of the external environment, internal conditions, and firm size on the DT of pharmaceutical companies. It can enrich the research on the DT of pharmaceutical companies in China.

The practical significance of this research is to provide suggestions for pharmaceutical companies to implement DT. The content include those as follows: (1) To realize strategic digitalization, senior managers of pharmaceutical companies should regard DT as a systematic project, carry out the overall planning, top-level design, and systematic promotion, establish a DT implementation team with the responsibility system of senior managers, and build an organization that supports the mechanisms and incentives of digital operations to ensure the implementation of DT; (2) to realize the digitalization of infrastructure, pharmaceutical companies should make full use of the new generation of information technology to promote the standardization of systems, interfaces, and network connection protocols of the hardware facilities, so as to enable the facilities of companies to have interconnection and security protection capabilities and form a foundation to support DT; (3) to realize the digitization of resources, pharmaceutical companies can build a digital platform and build a huge resource pool to support the company's efficient aggregation and dynamic allocation of various resources; (4) to realize the digitization of elements, pharmaceutical companies can use digital platforms to plan, store, and manage data resources in a unified manner to support data application innovation; (5) to realize business digitization, pharmaceutical companies can promote to reform and innovate the data-driven business processes such as drugs, R&D, clinical trials, production, operation management, marketing, and patient services and to form the new digital businesses and value-added space; and (6) to realize the benefits of digitalization, pharmaceutical companies can realize the value-added benefits and ecological construction in innovation and economic and social benefits.

### 6.2. Research Limitations

Due to the limitations of subjective and objective reasons, there are still some limitations in this research.

First of all, although this research initially has built the model of influencing factors of DT of pharmaceutical companies, the comprehensiveness of the model still has certain limitations. Secondly, the cross-sectional data were utilized to test the research hypotheses, but its disadvantage was that it cannot reflect the dynamic process of influencing factors on DT. Thirdly, there are limitations in data acquisition. This research adopted the method of purposive sampling and snowball sampling. Therefore, it is impossible to control the regions and objects involved in the data, which can weaken the persuasiveness of the research results to a certain extent.

## Figures and Tables

**Figure 1:** The theoretical framework of the DT of pharmaceutical companies.

**Figure 2:** The SEM model of influencing factors of pharmaceutical companies' DT.

**Table 1:** Demographic statistics.

Item	Category (*N* = 395)	Frequency	Percentage (%)
Position	General staff	183	46.33
	First-line manager	77	19.49
	Middle manager	45	11.39
	Senior manager	90	22.78

Region	Northeast	128	32.41
	East	98	24.81
	Central	103	26.08
	West	66	16.71

Age	Within 3 years	75	18.99
	Within 3–5 years	89	22.53
	Within 5–10 years	117	29.62
	More than 10 years	114	28.86

Size	Less than 100 people	47	11.90
	100–300 people	79	20.00
	300–2000 people	145	36.71
	More than 2000 people	124	31.39

Ownership type	State-owned enterprise	149	37.72
	Private enterprise	246	62.28

Situation of DT	No and there is no intention and plan for DT	25	6.33
	No but there is a willingness and plan for DT	66	16.71
	Yes, the DT project is in the early stage of construction	121	30.63
	Yes, the DT project has achieved certain results	183	46.33

**Table 2:** The validity of variables.

Variable	CR	AVE	Correlation of variables							
			CN	MC	GP	TT	DS	OC	LS	DT
CN	0.837	0.563	(0.750)							
MC	0.893	0.680	0.428^∗^^∗^	(0.824)						
GP	0.839	0.634	0.541^∗^^∗^	0.547^∗^^∗^	(0.796)					
TT	0.856	0.664	0.429^∗^^∗^	0.524^∗^^∗^	0.545^∗^^∗^	(0.815)				
DS	0.889	0.728	0.220^∗^^∗^	0.199^∗^^∗^	0.233^∗^^∗^	0.169^∗^^∗^	(0.853)			
OC	0.861	0.608	0.376^∗^^∗^	0.315^∗^^∗^	0.342^∗^^∗^	0.259^∗^^∗^	0.468^∗^^∗^	(0.780)		
LS	0.877	0.705	0.274^∗^^∗^	0.225^∗^^∗^	0.280^∗^^∗^	0.180^∗^^∗^	0.407^∗^^∗^	0.481^∗^^∗^	(0.839)	
DT	0.854	0.594	0.418^∗^^∗^	0.432^∗^^∗^	0.449^∗^^∗^	0.396^∗^^∗^	0.382^∗^^∗^	0.552^∗^^∗^	0.428^∗^^∗^	(0.771)

Notes: ^∗^^∗^*P* < 0.01. The square root of AVE is presented in parentheses.

**Table 3:** The fitting indexes of the models.

Fitting index	*χ * ^2^/df	RMR	RMSEA	GFI	AGFI	NFI	IFI	CFI	TLI
Reference value	<5	<0.1	<0.08	>0.8	>0.8	>0.8	>0.8	>0.8	>0.8
The overall CFA model	1.675	0.058	0.041	0.911	0.888	0.932	0.972	0.971	0.966
The second-order factor model of EE	4.16	0.088	0.09	0.899	0.857	0.927	0.944	0.943	0.929
The second-order factor model of IC	1.151	0.029	0.02	0.982	0.969	0.985	0.998	0.998	0.997
The SEM model of DT	1.858	0.163	0.047	0.896	0.876	0.92	0.962	0.961	0.957

**Table 4:** The correlation analysis of variables.

	Position	Region	Size	Age	Type	Action	CN	MC	GP	TT	DS	OC	LS	EE	IC	DT
Position	1															
Region	−0.097	1														
Size	0.045	−0.099	1													
Age	0.104^∗^	−0.091	−0.006	1												
Type	0.021	0.035	−0.024	−0.531^∗^^∗^	1											
Action	0.079	−0.169^∗^^∗^	0.009	0.668^∗^^∗^	−0.496^∗^^∗^	1										
CN	0.131^∗^^∗^	−0.053	0.057	0.051	−0.074	0.039	1									
MC	0.086	−0.075	0.151^∗^^∗^	0.172^∗^^∗^	−0.146^∗^^∗^	0.151^∗^^∗^	0.428^∗^^∗^	1								
GP	0.121^∗^	−0.125^∗^	0.075	0.098	−0.128^∗^	0.067	0.541^∗^^∗^	0.547^∗^^∗^	1							
TT	0.035	−0.075	0.111^∗^	0.06	−0.042	0.053	0.429^∗^^∗^	0.524^∗^^∗^	0.545^∗^^∗^	1						
DS	0.211^∗^^∗^	−0.093	0.052	0.119^∗^	−0.08	0.089	0.220^∗^^∗^	0.199^∗^^∗^	0.233^∗^^∗^	0.169^∗^^∗^	1					
OC	0.200^∗^^∗^	−0.064	0.041	0.109^∗^	−0.145^∗^^∗^	0.066	0.376^∗^^∗^	0.315^∗^^∗^	0.342^∗^^∗^	0.259^∗^^∗^	0.468^∗^^∗^	1				
LS	0.151^∗^^∗^	−0.091	0.097	0.169^∗^^∗^	−0.148^∗^^∗^	0.088	0.274^∗^^∗^	0.225^∗^^∗^	0.280^∗^^∗^	0.180^∗^^∗^	0.407^∗^^∗^	0.481^∗^^∗^	1			
EE	0.117^∗^	−0.105^∗^	0.125^∗^	0.121^∗^	−0.125^∗^	0.099	0.745^∗^^∗^	0.792^∗^^∗^	0.840^∗^^∗^	0.789^∗^^∗^	0.259^∗^^∗^	0.407^∗^^∗^	0.303^∗^^∗^	1		
IC	0.235^∗^^∗^	−0.103^∗^	0.079	0.165^∗^^∗^	−0.157^∗^^∗^	0.101^∗^	0.367^∗^^∗^	0.311^∗^^∗^	0.360^∗^^∗^	0.256^∗^^∗^	0.776^∗^^∗^	0.828^∗^^∗^	0.786^∗^^∗^	0.408^∗^^∗^	1	
DT	0.169^∗^^∗^	−0.157^∗^^∗^	0.216^∗^^∗^	0.199^∗^^∗^	−0.132^∗^^∗^	0.138^∗^^∗^	0.418^∗^^∗^	0.432^∗^^∗^	0.449^∗^^∗^	0.396^∗^^∗^	0.382^∗^^∗^	0.552^∗^^∗^	0.428^∗^^∗^	0.535^∗^^∗^	0.573^∗^^∗^	1

Notes: ^∗^*P* < 0.05, ^∗^^∗^*P* < 0.01, ^∗^^∗^^∗^*P* < 0.001.

**Table 5:** Parameter estimates for the model variables.

Hypothesis	Hypothesis path			Estimate	S.E.	C.R.	P	Standardized estimate
H1	DT	<---	EE	0.63	0.088	7.094	^∗∗∗^	0.43
H2	DT	<---	IC	0.95	0.117	8.081	^∗∗∗^	0.59

Notes: ^∗^*P* < 0.05, ^∗∗^*P* < 0.01, ^∗∗∗^*P* < 0.001.

**Table 6:** The results of common method biases test.

Component	Initial eigenvalue			Extraction sums of squared loadings		
	Total	Variance (%)	Cumulative (%)	Total	Variance (%)	Cumulative (%)
1	10.011	35.753	35.753	10.011	35.753	35.753
2	3.462	12.363	48.116	3.462	12.363	48.116
3	1.703	6.083	54.199	1.703	6.083	54.199
4	1.531	5.469	59.668	1.531	5.469	59.668
5	1.453	5.19	64.858	1.453	5.19	64.858
6	1.36	4.856	69.714	1.36	4.856	69.714
7	1.205	4.305	74.019	1.205	4.305	74.019
8	1.059	3.781	77.8	1.059	3.781	77.8
…						

**Table 7:** Results from the multiple regression analysis of EE on DT.

Independent variables		Dependent variable: DT						
		Model 1	Model 2	Model 3	Model 4	Model 5	Model 6	Model 7
Position	P2	0.161	0.081	0.098	0.071	0.105	0.043	0.053
	P3	0.303^∗^	0.103	0.301^∗^	0.17	0.228	0.132	0.155
	P4	0.383^∗^^∗^^∗^	0.254^∗^	0.282^∗^^∗^	0.247^∗^	0.33^∗^^∗^	0.227^∗^	0.213^∗^

Region	R2	0.251^∗^	0.115	0.163	0.18	0.173	0.1	0.114
	R3	0.067	−0.144	−0.02	−0.009	−0.053	−0.118	−0.127
	R4	−0.463^∗^^∗^^∗^	−0.24	−0.313^∗^	−0.208	−0.256^∗^	−0.164	−0.202

Age	A2	0.293	0.317^∗^	0.214	0.14	0.166	0.15	0.131
	A3	0.503^∗^^∗^	0.536^∗^^∗^^∗^	0.469^∗^^∗^	0.442^∗^^∗^	0.408^∗^	0.4^∗^^∗^	0.381^∗^
	A4	0.46^∗^	0.47^∗^^∗^	0.345^∗^	0.382^∗^	0.382^∗^	0.341^∗^	0.335^∗^

Type	T2	−0.056	−0.017	−0.01	0.037	−0.048	0.013	0.022

Action	Action2	−0.628^∗^^∗^	−0.497^∗^^∗^	−0.567^∗^^∗^	−0.411^∗^	−0.54^∗^^∗^	−0.451^∗^	−0.433^∗^
	Action3	−0.449^∗^	−0.401^∗^	−0.409^∗^	−0.244	−0.355	−0.291	−0.29
	Action4	−0.532^∗^	−0.425^∗^	−0.506^∗^	−0.311	−0.424^∗^	−0.351	−0.338

Size			0.163^∗^^∗^^∗^	0.125^∗^^∗^	0.155^∗^^∗^^∗^	0.141^∗^^∗^^∗^	0.135^∗^^∗^^∗^	0.153^∗^^∗^^∗^

CN			0.389^∗^^∗^^∗^					

MC				0.352^∗^^∗^^∗^				

GP					0.348^∗^^∗^^∗^			

TT						0.331^∗^^∗^^∗^		

EE							0.589^∗^^∗^^∗^	0.568^∗^^∗^^∗^

Zscore(Size) ^∗^ Zscore(EE)								0.104^∗^^∗^

F		5.325^∗^^∗^^∗^	10.420^∗^^∗^^∗^	10.523^∗^^∗^^∗^	10.968^∗^^∗^^∗^	9.662^∗^^∗^^∗^	14.438^∗^^∗^^∗^	14.374^∗^^∗^^∗^

*R * ^2^		0.154	0.292	0.294	0.303	0.277	0.364	0.378

Adjusted *R*^2^		0.125	0.264	0.266	0.275	0.248	0.338	0.352

D-W		0.277	0.559	0.552	0.545	0.514	0.688	0.694

Maximum VIF		6.878	6.903	6.882	6.982	6.907	6.924	6.928

Notes: ^∗^^∗^^∗^*P* < 0.001, ^∗^^∗^*P* < 0.01, ^∗^*P* < 0.05. EE = external environment.

**Table 8:** Results from the multiple regression analysis of IC on DT.

Independent variables		Dependent variable: DT					
		Model 8	Model 9	Model 10	Model 11	Model 12	Model 13
Position	P2	0.161	0.109	0.03	0.048	−0.001	0.012
	P3	0.303^∗^	0.177	0.058	0.21	0.042	0.047
	P4	0.383^∗^^∗^^∗^	0.224^∗^	0.125	0.234^∗^	0.083	0.09

Region	R2	0.251^∗^	0.166	0.025	0.128	0.017	−0.001
	R3	0.067	0.026	−0.058	−0.021	−0.052	−0.06
	R4	−0.463^∗^^∗^^∗^	−0.326^∗^	−0.283^∗^	−0.289^∗^	−0.235^∗^	−0.263^∗^

Age	A2	0.293	0.236	0.245	0.259	0.213	0.201
	A3	0.503^∗^^∗^	0.44^∗^^∗^	0.458^∗^^∗^	0.401^∗^	0.338^∗^	0.323^∗^
	A4	0.46^∗^	0.408^∗^	0.395^∗^	0.333^∗^	0.308^∗^	0.286

Type	T2	−0.056	−0.024	0.084	−0.009	0.049	0.056

Action	Action_2	−0.628^∗^^∗^	−0.479^∗^	−0.482^∗^^∗^	−0.486^∗^	−0.404^∗^	−0.397^∗^
	Action_3	−0.449^∗^	−0.376	−0.314	−0.293	−0.248	−0.239
	Action_4	−0.532^∗^	−0.418	−0.333	−0.347	−0.263	−0.243

Size			0.156^∗^^∗^^∗^	0.161^∗^^∗^^∗^	0.142^∗^^∗^	0.145^∗^^∗^^∗^	0.149^∗^^∗^^∗^

DS			0.297^∗^^∗^^∗^				

OC				0.461^∗^^∗^^∗^			

LS					0.337^∗^^∗^^∗^		

IC						0.622^∗^^∗^^∗^	0.639^∗^^∗^^∗^

Zscore(Size) ^∗^ Zscore(IC)							0.092^∗^^∗^

*F*		5.325^∗^^∗^^∗^	8.773^∗^^∗^^∗^	16.834^∗^^∗^^∗^	9.842^∗^^∗^^∗^	16.381^∗^^∗^^∗^	16.113^∗^^∗^^∗^

*R * ^2^		0.154	0.258	0.4	0.28	0.393	0.405

Adjusted *R*^2^		0.125	0.228	0.376	0.252	0.369	0.38

D-W		0.277	0.435	0.771	0.492	0.686	0.67

Maximum VIF		6.878	6.917	6.926	6.965	6.969	6.979

Notes: ^∗^^∗^^∗^*P* < 0.001, ^∗^^∗^*P* < 0.01, ^∗^*P* < 0.05. IC = internal conditions.

**Table 9:** Summary of research hypotheses.

Hypothesis	Validation results
H1: The external environment can have a significant influence on the DT of pharmaceutical companies	Supported
H1a: Customer needs can have a significant influence on the DT of pharmaceutical companies	Supported
H1b: Market competition can have a significant influence on the DT of pharmaceutical companies	Supported
H1c: Government policy can have a significant influence on the DT of pharmaceutical companies	Supported
H1d: Digital technology can have a significant influence on the DT of pharmaceutical companies	Supported
H2: The internal conditions can have a significant influence on the DT of pharmaceutical companies	Supported
H2a: Digital strategy can have a significant influence on the DT of pharmaceutical companies	Supported
H2b: Organization capability can have a significant influence on the DT of pharmaceutical companies	Supported
H2c: Leadership can have a significant influence on the DT of pharmaceutical companies	Supported
H3: Firm size can have a significantly regulatory influence on the relationship between the external environment and the DT of pharmaceutical companies	Supported
H4: Firm size can have a significantly regulatory influence on the relationship between the internal conditions and the DT of pharmaceutical companies	Supported

## Data Availability

The data used to support the findings of this study are included within the article.
